The article "Implementation of organization and end-user computing-anti-money laundering monitoring and analysis system security control" was retracted in 2025. Reasons: compromised peer review; unreliable results or conclusions; concerns about the peer review; concerns about the article.

# Implementation of organization and end-user computing-anti-money laundering monitoring and analysis system security control

**DOI:** 10.1371/journal.pone.0258627

**Published:** 2021-12-09

**Authors:** Ling Sun

**Affiliations:** School of Economics and Management, Nanjing Institute of Industry Technology, Nanjing, Jiangsu, China; Qingdao University, CHINA

## Abstract

The Monitoring and Analysis Centre for the fight against money laundering is a valid financial information body which is responsible for collecting, analysing and providing financial information and conducting international exchanges of financial information for relevant undertakings. By constructing the analysis of the monitoring of the local and foreign currency and of the data transmission subsystem in the plan for the transitional period against In the light of the above, the Commission will continue to monitor the implementation of the acquis in the light of the progress made in implementing the acquis future new systems. The purpose of this paper is to study the research and implementation of the security control of the anti-money laundering monitoring and analysis system. This article studies the application of decision tree analysis technology in the anti-money laundering monitoring system of insurance companies to achieve the purpose of improving the anti-money laundering monitoring technology and capabilities of insurance companies. The emergence of data mining technology provides a new system solution for anti-money laundering monitoring. For insurance anti-money laundering, how to find potential money laundering cases in suspicious and large surrender transactions is key. The experimental data show that the decision tree method is the best predictor of the customer category between the insurance application and the surrender days. The decision tree analysis technology has greatly improved the security monitoring capabilities of the insurance in the anti-money laundering monitoring system. Experimental data shows that the security control capabilities of the anti-money laundering monitoring and analysis system make the accuracy of the entire model reach 95%, the accuracy of large and suspicious transactions reaches 88.6%, and the correct classification of customers is about 99.6%.

## Introduction

With the strong development of the financial sector, the financial sector of my country is facing more security risks [1]. Among them, money laundering crimes develop in various ways from illegal activities introduced into the financial system and cause rapid damage to the country and society. All kinds of capital-based criminal activities are a shadow of its development. As an economic crime, money laundering has become the third largest trading activity in the world after foreign currency and oil, with a very rapid growth rate. It poses a serious threat to the national security of all countries and poses a threat to the development of the world economy.

Decision tree algorithm is the most widely used method in data mining classification algorithms. This is mainly because the decision tree algorithm has obvious advantages over other algorithms. The advent of data mining technology has given a new direction to monitoring against money laundering. In the easiest way to monitor, if you can use the last word of the technology to provide support to the Department of Legal Insurance for income from illegal activities, will significantly improve the effectiveness of the anti-money laundering project of insurance companies. For insurance against the legalisation of income from illegal activities, how to find possible cases of legalisation of income from illegal activities in suspect and large Delivery transactions are the key.

Scholars such as Helmy T H think that money laundering is a global problem that affects all countries to varying degrees. Although many countries accept money laundering, in the long run, foreign crime "money laundering will attract crime" [2]. Criminals will first inspect a country, establish a network and finally locate their criminal activities there. Most financial institutions have an anti-money laundering solution (AML) in place to combat investment fraud. The powerful anti-money laundering system of any financial institution mainly depends on a properly designed and effective monitoring system [3]. The main purpose system of AML monitoring is to identify potentially suspicious behavior embedded in legitimate transactions. Scholars such as Helmy TH use various technologies to enhance the surveillance framework of surveillance functions. This framework depends on rule base monitoring, behavior detection monitoring, cluster monitoring and monitoring based on link analysis [4]. Soudijn M R J and other scholars analyzed four types of Dutch crime models in money laundering reports. These reports are part of a four-year cycle that regularly outlines organized crime in the Netherlands. Tighter anti-money laundering laws and greater awareness of the profits of organized crime, and subsequent attention to the profits of organized crime, have led to increasing confiscation and conviction of money laundering. Although the analysis of crime patterns in money-laundering reports is not suitable for studying the effects of displacement or other changes (lack of precise data), they can be used as a tool for comparison and further policy research. Scholars such as Soudijn M R J found that some changes have taken place in money laundering methods and new convenience tools. Technology is the biggest driving force behind identified changes [5]. However, it turns out that the same method of money laundering has continued to prevail over the years. In this case, no innovation can be found. Even with the advent of digital opportunities and cryptocurrencies, cash is still widely used. Scholars such as Soudijn M R J found that the continuity of money laundering methods indicates that the risk of detection is very low or the consequences are negligible. These studies have a certain reference value for this paper, but due to the lack of experimental samples, it is difficult to copy in practice and does not have a universal role.

Currently, the latest technology lags behind the illegal registration of money from illegal activities in the insurance sector and advanced mining technology is not being used; information about. This article explores the use of wood analysis technology to determine the legitimacy of the revenue system from the illegal activities of insurance companies in order to improve legal technology to assess the illegal activities and income of insurance companies. In accordance with certain laws and regulations against the illegal registration of proceeds from illegal activities, this document uses data analysis and uses examples to create a model for extracting information that is consistent with a license to insure money from illegal activities [6]. companies. Improvement of information on the creation of appropriate operating systems or the conduct of existing operations, and the use of funds in the insurance business to assess the risk of misuse, have eliminated the effectiveness and effectiveness of the fight against money laundering.

## Programs method

### Security policy

The security policy system has always been the political soul and the technical core of maintaining the security of information and international network communication systems. It is the sum of the names of any set of relevant laws, regulations and protective measures that an undertaking has taken to protect the release, the management and use of sensitive corporate information and data resources. Security policies should be considered from three basic levels:

#### Abstract security policy

A security policy can usually be expressed as a series of technical documents described in the natural language. It is an analysis and development of network companies based on their own business, cyber threats and potential risks, as well as higher management systems and laws. A set of basic rules that come out to limit which network resources should be used by network users and how to use these resources correctly [7, 8].

#### Global Automatic Security Policy (GASP)

It consists primarily of a subset of the Agency’s abstract security policy and specific management organisation rules and policy constraints established by: the organisation and can be designed and applied automatically by other computers, routers and other electronic devices. Security that cannot be applied automatically by other computers Policies are applied automatically by other technical means such as environmental security, such as safety management systems. The global automatic security policy is mainly considered from various aspects of security protection functions, and is divided into information identification and security authentication protection policies, authorization and access control protection policies, information security confidentiality and data integrity protection policies, digital signatures and data anti-virus repudiation protection Strategy, security data audit protection strategy, intrusion data detection protection strategy, response and data recovery protection strategy, virus attack prevention protection strategy, fault tolerance and data backup protection strategy, etc. [9].

#### Local execution strategy (LESP)

It is usually a subset of the CFSP network distributed between the terminal network management system, the relay management system and other implementation systems. The sum of all entities and the number of LESPs in the network are a specific CFSP application. Partially enforceable security policy rules are a form of locally enforceable security regulations and enforceable security rules that can be applied by local elements of physics. System and local elements of a logical system, such as natural access code management policies, security wall filtering management rules, Identity control management system elements in the identity control management system include security identity control management policies, access control; and Application topic access tables, associated resource access control lists and security policy labels on system elements [10].

### Security access control scheme

Advanced users of the system can usually directly access all data on the virtual host, database or other related network media without using any designated network application software, using network commands or other network-assisted management software, and access control is targeted at this type. Designed by users [11]. Security access control technology is the main technical strategy for preventing the security risks of national networks and protecting the network. It is not only to ensure that the national network’s information resources are not used or have no illegal and malicious access. Significant technical resources. The main types of access control solutions currently used in this AML system security check are:

#### User authentication control

Designed for application-level users, including user management, user authentication, and user authorization:

User profile management mainly includes enterprise user profile management and maintenance, user identity authentication, and registration and authorization process management [12]. The system management user must first register for user login system authentication before being allowed to operate using the corresponding system business management functions. System management users are generally divided into a management system user and other operating system users. The management system user generally refers to the system management operator, while the management operating system user generally refers to the user data analysis manager or System approval manager.

#### User authentication method

User authentication uses user name + password + smart card authentication. Since the user name and password need to be remembered, need to be transmitted on the physical line and remain unchanged for a certain period of time, this method also has the possibility of malicious misappropriation. However, since the system is based on the intranet at this stage, risks are avoided to a minimum [13].

#### User authorization

If the user passes the identity authentication, it does not mean that he can access any resource of the system, and he must also authenticate the resource authority. The system mainly needs to deal with the following in the user authority authentication:

An application provided by the service system; logical components in the object Java server; various information content of the resource system; operating a specific action; the entity that the user performs the operation, the owner of the permission; a collection of several permissions for the role. Users can belong to multiple roles or not to any role.

#### Network access control

After determining the user authentication control, the first layer of access control is the access control to the network. You can control the user’s network access time, available network resources, and access ports based on user permissions. User network access control can be divided into three steps: user name identification and verification, user password identification and verification, and default checking of user accounts [14].

#### Database security

Including database backup and recovery, database user role management. Here mainly describes the database user role management scheme. The basic measures taken by database systems in using roles to manage database security are:

By verifying the username and password, prevent illegal users from entering in the database and from accessing the database illegally. granting users certain authorisations to restrict users from operating the database to allow users access to perform underlying entities data to prevent users from accessing unauthorised data; Provide database entity access auditing mechanism, so that the database administrator can monitor the data access situation and system resource usage in the database; use the view mechanism to restrict access to the base table row and column set [15, 16]. The basic strategy of role management is to classify all clients according to the nature of work and grant different user roles to each user; to different user roles, grant different database object access permissions according to the data source they use.

#### Network monitoring and lock control

The Network Manager shall monitor the network and the server shall record the user’s access to any network resource in real time. When unlawful access to the network is detected during network monitoring, the server shall be able to issue a warning in the form of text, graphics or sound and shall inform: the Network Manager [17]. When the system detects illegal access to an account multiple times, the web server should be able to automatically lock the account and submit relevant information to the upper-level application. Fig 1 is a flowchart of security information verification.

**Fig 1:** Safety information verification flowchart.

### Related theories of decision tree analysis

The advent of data mining technology has provided a new direction for anti-money laundering monitoring. In the easiest way to monitor, if the latest technology can be used to provide support to the insurance anti-money laundering department, it will greatly improve the efficiency of insurance companies’ anti-money laundering work [18]. For insurance anti-money laundering, how to find potential money laundering cases in suspicious and large surrender transactions is key.

#### General generation process of decision tree

First, use the training set to build an original decision tree model. Second, pruning the original decision tree model. Pruning can reduce the interference effect caused by the noise in the training set. The following is the decision tree generation algorithm and simplified flowchart shown in Fig 2.

**Fig 2:** Decision tree generation algorithm and simplified flowchart.

#### Classification of decision trees

According to the different branching schemes of decision trees, they can be divided into three categories: algorithms based on information theory methods, algorithms based on chi-square distribution indicators, and algorithms based on minimum GINI indicator method [19].

1. The algorithm representatives of the information theory method are: ID3, C4.5;
2. The indicators based on the chi-square distribution index algorithm are: CHAID, QUEST;
3. Algorithms based on the minimum GINI indicator method are CART and SLIQ.

#### Algorithm of decision tree

The theory of entropy and information theory The definition of entropy in information theory is: Any system has a state function, which can be defined as entropy [20]. In information theory, entropy and information are opposite. Entropy is a measure of the arbitrariness and uncertainty of the system. Information is a measure of order and certainty. So the information is also called negative entropy. Information Entropy is defined as:

$$\mathrm{Entropy}(p_{1},p_{2},\ldots .p_{n})=-p_{1}\log_{2}p_{1}-p_{2}\log_{2}p_{2}\ldots -p_{n}\log_{2}p_{n}$$ (1)

$$I\mathrm{nfo}(S)=\mathrm{Entropy}(p_{1},p_{2},\ldots ,p_{n})=\sum_{i=1}^{n}p_{i}\log_{2}p_{i},(1\leq i\leq n)$$ (2)

$$\mathrm{gini}(T)=1-\overset{n}{\underset{i=1}{\sum }}p^{2}$$ (3)

In the specific classification process, the sample set T is divided into T1, T2, A is the number of samples in T, A1 is the number of samples in T1, and A2 is the number of samples in T2. The gini coefficient for this classification is:

$$\mathrm{gini}(A)=\frac{A_{1}}{A}\mathrm{gini}(A_{1})+\frac{A_{2}}{A}\mathrm{gini}(A_{2})$$ (4)

$$X^{2}=\overset{J}{\underset{J=1}{\sum }}\overset{I}{\underset{i=1}{\sum }}\frac{{\left(n_{ij}-m_{ij}\right)}^{2}}{m_{ij}}$$ (5)

Among them,

$$n_{ij}=\sum_{n}f_{n}I(x_{n}=i\Lambda y_{n}=j)$$ (6)

$$p=P_{r}(x_{d}^{2}>X^{2})$$ (7)

d=(J−1)(I−1) (8)

$$\bar{y}=\frac{\sum_{n\in D}w_{n}f_{n}y_{n}}{\sum_{n\in D}w_{n}f_{n}}$$ (9)

$$p=P_{r}(F(I-1,N_{f}-I)>F)$$ (10)

*CART algorithm*. CART is based on the Gini coefficient. The specific method is to split the currently selected sample set into two sub-sample sets, and each child node of the generated decision tree has two branches [21]. Therefore, the decision tree generated by the CART algorithm is a simple binary tree. The CART algorithm is based on the minimum distance Gini Index standard. When the CART algorithm is used, the majority voting method is used. When the distribution of the sub-datasets at the nodes of a branch in the generated decision tree basically belongs to a class, the majority records the class of the node is used as the class identifier of the node. Stop generating decision trees for the node, and the node becomes a leaf node. Repeat the above process until the final decision tree meets the requirements.

*CHAID algorithm*. The CHAID algorithm is a kind of chi-square statistics. It is a classification method that establishes a decision tree by determining the best segmentation. This algorithm uses the dependent variable as the root node to classify each independent variable and calculate the chi-square value of the classification. If the classification of multiple independent variables is significant, compare the significance of these classifications by the P value, and use the most significant classification as the child node. This method can automatically merge the categories in the independent variables to maximize the significance [22].

*QUEST algorithm*. The QUEST algorithm mainly involves the determination of branch variables and segmentation values, but the choice of the two is handled according to different strategies. When determining branch variables, the independence of each attribute variable to the target variable is tested separately. If the attribute variable is categorical, the chi-square test is used; if the attribute variable is distant, the F test is used. If there are significant differences in the means, the 2-Means clustering method is used to cluster the samples into two categories, including the initial extreme centers of the two extreme means, so that the target variable values are merged into two categories [23, 24].

### Predictive control method of nonlinear monitoring system

In nonlinear predictive control, the predictive model is nonlinear.


$$X_{k+1}=F(X_{k},U_{k}),X_{k}\in R^{n},U_{k}\in R^{n}$$ (11)

*X*_*k*_,*U*_*k*_ is the system state and system input at k time, respectively. Non-linear function:

$$F(•):R^{n}\times R^{m}\to R^{n}$$ (12)

Assuming that the system can be stabilized, the state and input satisfy the constraints:

$$\{\begin{array}{c} X_{k+i+1}\in X\\ U_{k+i+1}\in U,i\geq 0 \end{array}$$ (13)

X and U are the set including the origin. Let *X*_*k*+*i*+1_ and *U*_*k*+*i*+1_ be the predicted value of the state and input at time k at time k+1 in the future, where the state prediction equation is:

$$(\{\begin{array}{c} X_{k+i+1|k}=F(X_{k+1|k},U_{k+i|k}),i\geq 0\\ X_{k|k}=X_{k} \end{array}$$ (14)

Finite time domain predictive control usually selects quadratic performance indicators:

$$\underset{U_{k}}{\min}J_{N}(X_{k})=\sum_{i=0}^{N-1}\left({\left\|X_{k+1k}\right\|}_{Q}^{2}+{\left\|U_{k+1k}\right\|}_{R}^{2}\right)+{\left\|X_{k+Nk}\right\|}_{P}^{2}$$ (15)

$$X_{k+i+1|k}\in X,U_{k+i+1|k}\in U,i=o,1,\ldots ,N-1$$ (16)

or:

$$\underset{U_{k}}{\min}J_{N,M}(X_{k})=\sum_{j=0}^{M-1}{\left\|U_{k+j|k}\right\|}_{R}^{2}+\sum_{i=1}^{N}{\left\|U_{k+1|k}\right\|}_{Q}^{2}$$ (17)

$$\{\begin{array}{c} X_{k+i+1|k}\in X,U_{k+i|k}\in U\\ U_{k+s+M|k}=U_{k+M-1|k},s=0,1,\ldots ,N-M-1 \end{array}$$ (18)

Where N is the prediction time domain, M less than or equal to N is the control time domain, matrix Q is greater than or equal to 0, R greater than 0 is a symmetric matrix, and for any variable and non-negative matrix W, there is$\|\partial {\|}_{W}^{2}=\partial^{T}W\partial$. At each time k, the decision variables of the optimization problem are:

$$\{\begin{array}{c} U_{k}^{N}={\left[U_{k|k}^{T},U_{k+1|k}^{T},\ldots ,U_{k+N-1|k}^{T}\right]}^{T}\\ U_{k}^{M}={\left[U_{k|k}^{T},U_{k+1|k}^{T},\ldots ,U_{k+M-1|k}^{T}\right]}^{T} \end{array}$$ (19)

If the prediction time domain and control time domain of predictive control are both, the predictive control at this time is called infinite time domain predictive control = control. Its basic feature is that the objective function is the sum of an infinite time positive definite function, and the performance index is usually expressed for:

$$\underset{U_{k}}{\min}J_{\infty }(X_{k})=\sum_{i=0}^{\infty }\left({\left\|X_{k+1|k}\right\|}_{Q}^{2}+{\left\|U_{k+1|k}\right\|}_{R}^{2}\right)$$ (20)

$$X_{k+i+1|k}\in X,U_{k+i+1|k}\in U$$ (21)

The decision variables of optimization problem (20) at each moment are:

$$U_{k}={\left[U_{k|k}^{T},U_{k+1|k}^{T},\ldots \right]}^{T}$$ (22)

Due to the non-linear characteristics of the system (11), non-linear predictive control will inevitably be more difficult than linear predictive control in both theoretical analysis and practical application. The current theoretical research on nonlinear predictive control mainly focuses on several aspects such as stability, robustness and online calculation [25].

### Characteristics of money laundering

The particularity of money laundering is to prevent the flood of money laundering activities, which must be strictly stopped. The first step in combating money laundering is to properly identify money laundering crimes. Generally, money laundering has the following characteristics:

1. Various ways to make money. Due to the variety of sources of crime, money launderers often use post-money laundering methods to avoid surveillance and prosecution. In addition, money laundering has a long history: money laundering criminals have developed various methods of money laundering in order to avoid stricter supervision and penalties for money laundering, which has led to many difficulties in the field. Traditional methods of money laundering include the use of casino labels for trade, the purchase of artifacts and antiquities. As the deepening economic depth and ever-evolving internet information technology are also double-edged swords, this will provide more space for money laundering activities such as spectacle companies and fake business papers. Most importantly, a professional money laundering organization has now been set up to carry out the growing campaign of money laundering. They are mainly organized by many professionals and combine various means and methods of money laundering. Among them, it uses sophisticated financial instruments to conduct complex financial transactions through money laundering (such as Bitcoin).
2. The hidden nature of money laundering. It is easy to intuitively understand common crimes, that is, direct or indirect victims, and the consequences of the crimes or the damage they cause. However, money laundering crimes are different because specific criminal procedures are very hidden, the outcome of the crime or the danger of the crime cannot be intuitively understood, and there are no directly identifiable victims of money laundering crimes, so it is difficult to attract people’s attention. Because most governments control money laundering, financial institutions report transactions to authorities in excess of a certain amount (usually required by law). To avoid oversight, one approach is to "round up" large amounts of money to zero. Deposit funds into multiple accounts opened in the name of others, these accounts are not linked, and then transferred to the offender’s name through remittances, checks, etc.
3. The professional and technical nature of money laundering crimes. With financial marks, financial crimes have professional characteristics. Today, money laundering has become a very complex professional industry. Because the money laundering process is complex and often involves the financial and legal systems of different countries, only professionals who are familiar with the legal system and financial operations of each country can do so. It is usually managed by a team, or assisted by professional financial and legal personnel to obtain high profits.
4. Money laundering is transnational in nature. Although laws and regulations to combat money-laundering crimes exist in different countries, differences in financial transactions and legal systems in different countries have caused difficulties in international cooperation, which also provides opportunities for criminals. At present, many money-laundering crimes are usually transnational operations, and even use certain countries or regions to open confidential accounts or companies, such as Switzerland, the world’s largest offshore financial center, and the Swiss bank’s privacy system can also bypass the monitoring of audit institutions to some extent.

## Experiments

### Experimental settings

The research and implementation of the anti-money laundering monitoring and analysis system security control is to calculate the indicators that reflect the characteristics of customers or accounts, and is the basis for rule monitoring. From a calculation perspective, indicators are designed as basic indicators and rule indicators. Basic indicators are calculated directly from business data (mainly anti-money laundering related transaction data), while calculation rule indicators are mainly calculated from basic indicators. Therefore, the specific calculation of each indicator is performed step by step.

The characteristics of large and suspicious transactions of insurance companies include premium premiums. In long-term insurance, premiums are relatively high. Money launderers have sufficient illegal income in their hands and want to withdraw funds in a short time. Means, the author believes that the choice of payment method is likely to affect the type of customer, but this variable is not involved in the current large and suspicious transaction reports. Each period of independent variable premiums is divided into two groups, "0" means that each period of premiums is less than or equal to 10,000 yuan. "1" means that the premium per period is greater than 10,000 yuan. As the subject of financial crime is becoming highly educated, in order to avoid paying attention to intercourse, the overdue payment should also be taken seriously. The 10,000 yuan chosen here is mainly based on the average level of interim delivery.

The independent policy categories are divided into three groups. The company’s business types are accident insurance, property insurance and liability insurance. Therefore, "0" represents accident insurance, "1" represents property insurance, and "2" represents liability insurance. The independent variable insurance and surrender days interval is divided into three groups, 0 "means that the insurance and surrender days interval is greater than 100 days," 1 "means that the insurance and surrender days interval is less than 20 days, and" 2 "means the insurance and surrender days interval Between 20 and 100 days. Due to the limited number of money laundering transactions and the difficulty of obtaining national data, it is not possible to analyze the interval between the days of insurance and withdrawal. This article believes that money launderers are generally unwilling to spend too much time Withdraw funds, so the interval between insurance and surrender days is likely to be one of the variables to determine the type of customer. Here, any period between 20 days and 100 days is selected as the cutoff point. The accuracy of the model, the amount and accuracy of suspicious transactions, and the correct classification of customers are shown in Table 1.

**Table 1:** Extremely long intervals between insured and surrendered days.

Node	Node Cases	Node Percentage	Number Of Target Classification Node Cases	Target Classification Percentage
14	194	0.2%	162	30.2%
13	228	0.2%	52	9.7%
12	5195	5.0%	262	48.8%
10	1048	1.0%	21	3.9%
9	1141	1.1%	10	1.9%

### Experimental data and parameters

The research data of the anti-money laundering monitoring and analysis system security control research in this paper includes 1 dependent variable and 7 independent variables. These variables are identified as groups. The dependent variable is the customer category, that is, whether it is a large amount and a suspicious transaction user (bad and good users respectively; represented by 1,0). The independent insured person’s gender is divided into two groups, male and female, which are represented by "0" and "1", respectively. The purpose of this independent grouping is to determine whether the insured’s gender affects the type of customer. The independent insured person’s age range is divided into three groups, "0" means the insured person’s age is between 0–35 years old, "1" means the insured person’s age is between 36–55 years old, and "2" means the insured person’s age Over 55 years old. Because the statistics of people’s anti-money laundering are limited, the age distribution of money laundering molecules cannot be obtained. The payment method of independent variable is divided into payment (one-time payment) and period payment (payment by installments), which are expressed by "0" and "1" respectively. The characteristics of large and suspicious transactions of insurance companies include premium premiums. In long-term insurance, premiums are relatively high. Money launderers have sufficient illegal income in their hands and want to withdraw funds in a short time. Means, this article believes that the choice of payment method is likely to affect the type of customer, but this variable is not involved in the current large and suspicious transaction reports. The independent premium of each variable is divided into two groups, "0" means that the premium of each period is less than or equal to 10,000 yuan, and "1" means that the premium of each period is greater than 10,000 yuan. As the subject of financial crime is becoming highly educated, in order to avoid paying attention to intercourse, the overdue payment should also be taken seriously. The 10,000 yuan chosen here is mainly based on the average level of interim delivery.

The independent policy types are divided into three groups. The company’s business types are accident insurance, property insurance and liability insurance. Therefore, "0" represents accident insurance, "1" represents property insurance, and "2" represents liability insurance. The independent variable insurance and surrender days interval is divided into three groups. "0" indicates that the insurance and surrender days interval is greater than 100 days, "1" indicates that the insurance and surrender days interval is less than 20 days, and "2" indicates the insurance and surrender days. The interval is between 20–100 days. Because the number of confirmed money laundering transactions is limited and it is difficult to obtain data nationwide, it is impossible to make a relevant analysis of the interval between the days of insured and surrender. Money launderers are generally reluctant to spend too much time withdrawing funds, so the interval between insured and surrender days is likely to be one of the variables to judge the type of customer. Here we choose 20 and 100 days as the cut-off point. As shown in Table 2.

**Table 2:** Preprocessing data table.

	Gender	Age	Insurance Amount	Payment Mode	Premium Per Period	Type Of Policy	Insurance And Surrender Days Interval	Customer Type
1	1	0	0	0	0	0	0	0
2	0	0	0	1	0	1	0	0
3	1	0	0	1	0	0	2	0
4	1	0	0	1	0	0	2	0
5	1	0	0	0	0	0	2	0

## The discussion

### Model analysis

(1) In this example, there is only one target classification, so the node table has only one gain. Nodes represent the total number of cases at each endpoint, and node percentage is the total number of cases at each node divided by the total number of cases at the root node. In this case, since the large and suspicious transaction objects were selected as the categories of interest, the gain represents the number and percentage of cases with large and suspicious transactions. For categorical dependent variables, the penultimate column is the percentage of cases in the target classification. The interest in this example is large and suspicious transaction objects, so the percentages of the endpoints of the target classification are shown in the table above. An index value greater than 100% indicates that the percentage of the target classification of each endpoint is greater than the percentage of the target classification of the root node. Conversely, when the index value is less than 100%, it means that the percentage of the target classification of each endpoint is less than the percentage of the target classification of the root node. The figure obtained is shown in Table 3 and Fig 3.

**Fig 3:** Percentage of target classification for each endpoint.

**Table 3:** Percentage of target classification for each endpoint.

Total Number Of Cases	Model Accuracy	Large And Suspicious Transactions	Classify Customers Correctly
**Classification**	100%	96%	90%
**Data 1**	100	96	0

(2) This article provides most practical tree diagram information in the form of a table. For each node, Table 3 shows the model tree table of CART: it includes the number and percentage of cases of the dependent variable in each classification. More important is the prediction classification of the dependent variable. According to the seventh column, only when the proportion is less than 0.2%, this customer is a large and suspicious transaction object. The 9th column represents the parent node, there are no other child nodes under node 1, nodes 3 and 4 are the parent nodes of node 2, node 5 and 6 are the parent nodes of node 3, and so on. Arguments are used to divide nodes. For example, nodes 1 and 2 are divided by the insurance and surrender interval, nodes 3 and 4 are divided by the insured amount, nodes 5 and 6 are divided by the period premium payment, and nodes 7 and 8 are divided by the payment mode. The penultimate column is the significance level, and their values are less than 0.001 in the model. The segmentation value of the node in the last column, node 1 is the group with the insurance and surrender interval greater than or equal to 20 days, node 2 is the group with the insurance and surrender interval less than 20 days, and so on. The data is shown in Table 4. Figure shown in Fig 4.

**Fig 4:** CART model data graph.

**Table 4:** Number of CART models.

Node	Number Of Cases	Independent Variable	Saliency	Split Value
0	103146	99.50%	-	-
1	97947	99.90%	0.001	20–100
2	5199	91.60%	0.001	<20
3	5109	94.20%	0.002	< = 200000
4	90	35.70%	0.002	>200000

### Analysis of factors affecting information security

Based on the analysis of the revised conceptual model of the factors affecting the effectiveness of anti-money laundering supervision, the paper verifies that commercial banks.

The path relationship between different influencing factors of anti-money laundering has both direct and indirect effects. Then, through the analysis of the influencing factors between the influencing factors, the quantitative characteristics of its effects are obtained. The calculation results are shown in Table 4. It is not difficult to see that the four levels of influencing factors involved in the study will jointly affect the effectiveness of anti-money laundering in commercial banks. Among them, anti-money laundering laws and regulations, organizations, employees, and anti-money laundering computer systems, etc. There is a direct relationship between effectiveness; anti-money laundering supervision, internal control of anti-money laundering, anti-money laundering costs, leadership, monitoring methods and skills and other factors have an indirect effect on the effectiveness of anti-money laundering. In general, the most obvious impact on the effectiveness of commercial banks’ anti-money laundering is anti-money laundering laws and regulations and anti-money laundering costs. As shown in Table 5 and Fig 5.

**Fig 5:** List of calculation results of the effects of various factors on the effectiveness of commercial banks’ anti-money laundering.

**Table 5:** List of calculation results of the effects of various factors on the effectiveness of commercial banks’ anti-money laundering.

Project	Direct Effect	Indirect Effect	Total Effect
**Anti-Money Laundering Laws And Regulations**	0.614	-0.097	0.517
**Anti-Money Laundering Regulation**	0	0.124	0.124
**Anti-Money Laundering Internal Controls**	0	0.034	0.034
**Anti-Money Laundering Costs**	0	-0.529	-0.529
**Organization**	0.348	0.015	0.363
**Leadership**	0	0.048	0.048
**Employee**	0.176	0	0.176
**Anti-Money Laundering Computer System**	0.236	0	0.236
**Monitoring Methods And Techniques**	0	0.031	0.031

(2) The implementation methods and audit capabilities of security application systems vary widely. Many application systems do not need to log in, operate directly, and cannot track user operations. There are also some application systems that do not have audit log records. For these uneven application systems, two methods can be used for implementation. The first method is to conduct secondary development of the application system itself and enhance the auditing capability according to the application system security audit monitoring technical specifications. The second method is to use auditing. The agent model, based on the original application system, develops a set of security audit agent systems, deployed on the front end of the application system, and uses the middle-layer working mode to audit user actions by intercepting user operations. The monitoring system uses people as the core, audits as the means, and technology as the guarantee. It implements monitoring of various audit object logs, realizes the informationization and standardization of security audit work, guarantees the security operation of the industry intranet, and improves the security audit level and work efficiency. Case-by-case investigation provides strong technical support. The overall architecture of the monitoring system is logically divided into three levels: the centralized display layer, the core processing layer, and the access switching layer. The data flow of the monitoring system is not limited to the division of layers and modules, and the work requirements can be implemented across layers and modules. The analysis results of the conceptual model of influencing factors are shown in the figure and table. Compared with the initial conceptual model, each action path is significant. The goodness-of-fit indicators of the revised structural model are improved compared to the initial model, χ2 is reduced from 1133.251 to 970.106, which is not significant at the level of 0.05; the RMR value is reduced from 0.088 to 0.029, which is less than the lower limit of 0.05; the RMSEA value 0.000, less than 0.08; values of GFI, AGFI, NFI, RFI, IFI, TLI, CFI all exceed the minimum standard of 0.9; values of PGFI, PNFI, PCFI have increased, all of which are greater than the minimum standard of 0.5; χ2 / df from 1.177 Reduced to 1.000, which is less than the minimum recommended value of 3. On the whole, the degree of fit of the revised model is more ideal. Overall, as shown in Fig 6, Table 6.

**Fig 6:** Parameter estimation table for the modified conceptual model of influencing factors on the effectiveness of anti-money laundering regulation.

**Table 6:** Parameter estimation table for the modified conceptual model of influencing factors on the effectiveness of anti-money laundering regulation.

Action Path	Estimated Value	Standardization	Standard Deviation	Critical Ratio
**Anti-Money Laundering Effectiveness**	0.531	0.614	0.037	14.487
**Anti-Money Laundering Regulation**	0.441	0.578	0.034	13.126
**Internal Control**	0.475	0.522	0.044	10.723

### Status quo of anti-money laundering

It is difficult to estimate the losses caused by fraud in the financial industry, but the total amount is about trillions of dollars a year:

In general, no industry is immune to fraud risks, and financial services have always been one of the industries with the most fraud. As shown in Table 7 and Fig 7, the amount of fraud detection in most industries declined from 2016 to 2019, with the highest decline in high-tech industries, reaching 15%. However, fraud in the retail and consumer goods industry and the construction industry showed a double-digit increase.

**Fig 7:** Comparison of the number of fraud cases in various industries worldwide.

**Table 7:** Comparison of the number of fraud cases in various industries worldwide.

Industry	Consumer Goods	Financial Consumption	Telecommunications	Service	Building	High Tech
**2016**	44%	52%	45%	48%	34%	51%
**2019**	59%	49%	45%	44%	44%	39%
**Rate Of Change**	15%	-3%	0%	-4%	10%	-12%

It can be seen from the above introduction that financial institutions need to conduct comprehensive monitoring of financial fraud. Financial fraud requires a comprehensive analysis of a large amount of information, and backward manual management methods can no longer adapt. Only by relying on high-tech methods, combined with manual management, and improving the automation level and processing capabilities of analysis, can the accuracy and processing capacity of risk prediction be gradually improved. Timeliness.

### Test analysis of anti-money laundering detection and analysis system

In order to evaluate and verify the processing efficiency of anti-money laundering construction based on data mining, data mining was tested, and under the same environment, it was compared with the original implementation through stored procedures. Apply data mining and stored procedures to the same data set to implement the same business logic respectively, in which the implementation of the stored procedures has undergone certain optimization work such as SQL tuning. Take 2 d, 5 d, 10 d, 20 d, 30d, 50d transactions respectively for testing. The test result is shown in Fig 8.

**Fig 8:** Test results of detection analysis system.

According to the data analysis in the figure, under the same number of rules, as the amount of data increases, the time consumption of stored procedures and data mining is increasing, and basically shows a linear growth trend, but the rule-based processing method, The time growth rate is slightly smaller.

## Conclusions

1. The security control of the anti-money laundering monitoring and analysis system studied in this article is a critical part of security auditing. Application system log monitoring can further improve the application system security audit function and achieve effective supervision of various application system audit functions in real time. Analyze the audit status and assess the current security status. Through the log monitoring system, it is possible to collect key application system logs, summarize and correlate them, find out traces of violations or suspicious behaviors, facilitate incident accountability, and improve efficiency. In short, the application of system log monitoring technology meets the needs of deep security audits and provides a new way for event accountability.
2. During the construction and development of computer network systems, the security design of the system is critical. According to the system’s security requirements and system investment, appropriate security measures must be adopted to prevent system failure and resist external intrusion. The goal. This paper proposes system security strategies from six aspects, each of which can be designed as a security subsystem in the security design of the system, and can be implemented using different technologies. In short, a network that adopts a secret security policy is a truly secure network and a useful network.
3. In the experiment of the security control of the anti-money laundering monitoring and analysis system studied in this paper, the correlation between large amounts and suspicious transactions is modeled through the CHAID algorithm, CART algorithm and QUEST algorithm in the decision tree to obtain the identification factors that affect the results. In the end, it was found that the identification factors of the three models are similar, mainly including the four factors of the interval between the insurance and surrender days, the amount of insurance, the premium per period, and the payment mode. The factors that have never been involved, so these two factors can be added to the actual operation of the insurance company. In addition, the accuracy of the three models as a whole is higher, which indicates that this model is suitable for this problem. The accuracy of the overall prediction classification of the three decision tree models is high, but the accuracy of misclassifying large and suspicious transactions into customers with good credit is low. By setting the misclassification cost and setting the misclassification cost of the suspicious transaction object as a good credit user to N times the misclassification cost of the good credit user as a suspicious transaction object (N is any real number greater than 1), the prediction classification can be significantly improved The accuracy of the model ultimately makes the accuracy of the entire model reach 95%, and the accuracy of large and suspicious transactions reaches 88.6%.
